The article "3D Convolutional Neural Network Framework with Deep Learning for Nuclear Medicine" was retracted in 2023. Reasons: signs of a paper mill; compromised peer review; unreliable results or conclusions.

# 3D Convolutional Neural Network Framework with Deep Learning for Nuclear Medicine

**DOI:** 10.1155/2022/9640177

**Published:** 2022-07-16

**Authors:** P. Manimegalai, R. Suresh Kumar, Prajoona Valsalan, R. Dhanagopal, P. T. Vasanth Raj, Jerome Christhudass

**Affiliations:** ^1^Department of Biomedical Engineering, Karunya Institute of Technology and Sciences, Coimbatore, India; ^2^Center for System Design, Chennai Institute of Technology, Chennai, India; ^3^Department of Electrical and Computer Engineering, Dhofar University, Salalah, Oman

## Abstract

Though artificial intelligence (AI) has been used in nuclear medicine for more than 50 years, more progress has been made in deep learning (DL) and machine learning (ML), which have driven the development of new AI abilities in the field. ANNs are used in both deep learning and machine learning in nuclear medicine. Alternatively, if 3D convolutional neural network (CNN) is used, the inputs may be the actual images that are being analyzed, rather than a set of inputs. In nuclear medicine, artificial intelligence reimagines and reengineers the field's therapeutic and scientific capabilities. Understanding the concepts of 3D CNN and U-Net in the context of nuclear medicine provides for a deeper engagement with clinical and research applications, as well as the ability to troubleshoot problems when they emerge. Business analytics, risk assessment, quality assurance, and basic classifications are all examples of simple ML applications. General nuclear medicine, SPECT, PET, MRI, and CT may benefit from more advanced DL applications for classification, detection, localization, segmentation, quantification, and radiomic feature extraction utilizing 3D CNNs. An ANN may be used to analyze a small dataset at the same time as traditional statistical methods, as well as bigger datasets. Nuclear medicine's clinical and research practices have been largely unaffected by the introduction of artificial intelligence (AI). Clinical and research landscapes have been fundamentally altered by the advent of 3D CNN and U-Net applications. Nuclear medicine professionals must now have at least an elementary understanding of AI principles such as neural networks (ANNs) and convolutional neural networks (CNNs).

## 1. Introduction

The use of artificial intelligence (AI) in molecular imaging and nuclear medicine has gained considerable momentum and promises to be a disruptive, yet inventive, technology. Nuclear medicine has been using AI for many years, and the excitement surrounding AI in radiology obscures this fact (e.g., cardiac quantitative software packages). Artificial neural networks (ANN), DL, and ML have all recently seen significant advances, which has reignited interest in AI while also sparking controversy about the ethical and legal issues that come with using AI in health and medicine. In the midst of this conversation, a crucial aspect is often overlooked: As with any tool, the best way to use AI is up to the user.

The article "3D Convolutional Neural Network Framework with Deep Learning for Nuclear Medicine" was retracted in 2023. Reasons: signs of a paper mill; compromised peer review; unreliable results or conclusions.

In nuclear medicine and radiology, a wide array of machine learning and deep learning capabilities are available. At one end of the spectrum, for example, there may be a straightforward use of machine learning for quality assurance, business analytics, risk assessment, and basic classifications. Detected, localized, and classified images may be found in a wide range of deep learning applications. Another extreme is the large and complex CT, PET, and MRI data put into convolutional neural networks (CNNs) to get insight into segmentation, detection, localization, classification, quantification, and radiomic feature extraction using deep learning (DL). Certain CNN and deep learning applications may go beyond the extreme (ultra-zone) when used in conjunction with hybrid technologies that need picture registration across several modalities, equipment, and sample lengths. At the low end of the spectrum (dubbed the “infra zone”), the use of artificial neural networks (ANNs) and machine learning (ML) enables the study of both small and big datasets concurrently.

Clinical and scientific skills may be improved as well as workflow and productivity in nuclear medicine by using AI in molecular imaging and nuclear medicine. Innovation comes with a sense of duty to one's profession and to one's patients. Social, legal, and ethical duties all fall under this umbrella. Ethical, social, and legal concerns with AI in molecular imaging and nuclear medicine center on the data utilized, the algorithms employed, and the practical application of those algorithms.

As a result of technological advancements such as multimodality imaging equipment being deployed in the 2000s [1] and rapid detector technologies being developed [1, 2], nuclear medicine and radiology have seen significant progress in the previous two decades. Software advancements have also resulted in significant increases in signal-to-noise ratio and reconstructed picture spatial resolution, for example, by including information from the time of flight (ToF) and point-spread function into PET image reconstruction [3]. Nuclear medicine images are employed in a relatively restricted manner in the majority of clinical articles, clinical research, and, most importantly, in daily clinical practice (i.e., analyzed mostly visually or semiquantitatively). Medical image analysis is becoming increasingly automated, and many characteristics, some of which may not be visible to the untrained eye, are being extracted [4, 5]. When it comes to precision medicine, the most important goal of this paradigm shift is to effectively use the information offered by imaging investigations to influence patient treatment workflow. Medical imaging should play a larger and more essential role in this new paradigm than just diagnosing. It should also play a bigger and more important role in treatment planning, monitoring, and evaluation, as well as predictive modeling and stratification, to become an important part of the future clinical decision-making process.

The article "3D Convolutional Neural Network Framework with Deep Learning for Nuclear Medicine" was retracted in 2023. Reasons: signs of a paper mill; compromised peer review; unreliable results or conclusions.

The ANN is essential to MR and DL in nuclear medicine. An ANN is a node-based analytic technique that consists of many layers of nodes. Radiomic characteristics derived from the picture files or the photos themselves may be used as inputs to a CNN. Clinical and research capacities in nuclear medicine are being reengineered and reimagined by AI. An ANN is made up of nodes arranged in a hierarchical structure (depth). Inputs from other nodes are weighted (Figure 1). By modifying the node weightings, the ANN aims to maximize accurate outputs as assessed against a grounded truth [6, 7]. Iterations (epochs) of the answer get it closer to the truth.

The study of algorithms that learn and develop over the course of time is known as machine learning, and it is an essential concept in artificial intelligence. Unsupervised or (semi-) supervised learning is the most common classification. Unsupervised learning involves discovering patterns in unlabeled data, while supervised learning relies on labels to make inferences about categorization or regression, and semisupervised learning involves a small quantity of labeled data and a big amount of unlabeled data. When it comes to medical imaging, the typical procedure or the deep learning pipeline is often applied directly to the majority of tasks.

It is often believed that the advent of AI in medicine would lead to “superhuman” capabilities and more precise treatment. Conversely, it is easy to overlook the fact that a significant portion of a physician's daily work consists of routine tasks, and that delegating these tasks to AI would free up human resources to focus on higher value activities that typically necessitate human attributes like cognitive insight, creativity, empathy, or meaning.

### 1.1. Artificial Intelligence and Deep Learning Used in Nuclear Medicine Imaging

Artificial Intelligence (AI) has a broad range of potential applications in nuclear medicine [8]. Data processing at the detector level is the initial stage in using AI for picture reconstruction, including adjustments for the many physical processes involved in the detection process (e.g., attenuation and scatter). AI may be used for a variety of image processing tasks, including denoising, segmentation, and fusion, in addition to reconstruction. To wrap things up, artificial intelligence (AI) may be used to build models based on information gleaned from photos that can be utilized for predictive, tailored therapy.

The article "3D Convolutional Neural Network Framework with Deep Learning for Nuclear Medicine" was retracted in 2023. Reasons: signs of a paper mill; compromised peer review; unreliable results or conclusions.

The software used to make PET images has also improved a lot over the years. For example, time of flight (ToF) information and point spread function can now be used to make PET images look better. Some of the most important medical papers use nuclear medicine images very carefully. This is true for both clinical studies and “normal” medical care (i.e., analyzed mostly visually or semiquantitatively).

PET scanners with lots of crystal pixelation could use a computer network to improve picture resolution and noise quality, as well as to figure out the time of flight from two digitized detector waveforms that are both digitized at the same time [9, 10]. When it comes to iterative picture reconstruction, the use of a deep neural network may increase the final product's quality [11, 12]. For attenuation adjustment and registration in PET/MR and PET/CT, deep learning approaches have already been presented [13–17]. These methods can create attenuation maps with excellent accuracy. Deep learning, like the MLAA, has been used to enhance the maximum likelihood reconstruction of activity and attenuation in ToF PET data (MLAA) [18]. It is one of the most common ways to use deep learning to process images. Full-dose PET pictures are one example of how this technique may be employed [19] or how it can filter reconstructed PET images directly [20].

Images may be segmented and counted using an automated system. This can be used for diagnosis and treatment planning, among other things. Older, shaky machine learning frameworks could not attain the degree of automation and precision required for clinical practice or swiftly handle hundreds of radiomics patients simultaneously. A rising number of companies are depending on deep learning approaches to improve both automation and performance, although others are still using “older” techniques. Medical picture segmentation is an excellent use case for CNNs [21]. This may be explained by the fact that segmentation learning happens at the voxel level, as opposed to classification tasks (one label per picture) (one label per voxel). As a result, the network parameters may be trained more effectively. According to a recent PET functional volume segmentation MICCAI competition, a strategy using an already-trained CNN was the best (although not much higher than the results for some of the more traditional methods) [22]. Multiple PET/CT cosegmentation has been tackled using CNNs [23–25]. The radiomics pipeline is anticipated to give completely automated solutions for this stage, which will eliminate this key bottleneck, based on pipelines for tumor identification and segmentation that use a deep learning framework [26–28]. Planning, picture acquisition, analysis, and reporting are the four stages that make up a typical medical imaging workflow (Figure 2). The entrance and payment processes might also be incorporated. We have zeroed down on the steps of the process in which the doctor plays a pivotal role.

The article "3D Convolutional Neural Network Framework with Deep Learning for Nuclear Medicine" was retracted in 2023. Reasons: signs of a paper mill; compromised peer review; unreliable results or conclusions.

The fundamental concept that underpins the Mask R-CNN approach [29, 30] is to specialize an image classifier model by equipping it with a large number of trainable modules in order to extract features of varying sizes, bounding boxes, object classes, and individual masks.

Some of the datasets used for the analysis of nuclear imaging are as follows: MoNuSeg–Grand Challenge, Mitos-Atypia-14–Grand Challenge, Kaggle Data Science Bowl, dataset from immunohistochemistry, neurosphere dataset, and electron microscopy dataset.

## 2. Convolutional Neural Network

CNN uses convolution and pooling layers to extract features from pictures, but ANNs need particular data (features) to be fed into the system (Figure 3). A convolution approach employs a variety of kernels (often three by three) to apply to a subset array of pixels in an image in order to extract radiomic features, and the output of these kernels is summed together to generate a single integer value across all of the extracted features [31–35]. Before taking a sample from further in the convolution layers, activation functions form feature maps. Several layers of data are flattened as a consequence of several convolution, kernel, and pooling stages occurring in succession [32–34].

In order to extract radiomic information from photographs and offer an output as some sort of classification, convolutional and pooling levels are used in conjunction with a fully connected network in a CNN. Linear convolution is used to extract visual information from an input tensor by applying an appropriate kernel (often 3 × 3). Kernel elements are overlaid on input tensor elements, and the stride determines how often the kernel is moved. The kernel is applied to the input tensor one at a time, with a stride of 1. A stride of 2 is utilized when the kernel is applied to each and every second element of the input tensor. Down-sampling may be best saved for the pooling function if a stride bigger than 1 is used. One numerical value (and corresponding coordinate values) is generated by summating the product of the individual components of each input tensor and the kernel (output tensor). With the use of different kernels, each convolution layer may be created. However, the Z dimension is not compressed, despite the fact that it has been reduced in size.

The article "3D Convolutional Neural Network Framework with Deep Learning for Nuclear Medicine" was retracted in 2023. Reasons: signs of a paper mill; compromised peer review; unreliable results or conclusions.

Pooling is a technique for reducing the number of samples taken. There were two main ways to do this: global average pooling and max pooling. This is called “max pooling down.” It samples the components to get an output that is the same as the largest value in a certain area of data on the feature map. In order to do this, we down sample each group of four components until we get a single value for each that is the same as the maximum value. Global pooling makes the feature map into a 1 × 1 array with a single value for each element in this case. This makes the feature map easier to read. Mean value: The sum of the values of each element is equal to the sum of all the values of all of them. A single direction array of vectors is made from data that has been convolution and pooled (numbers).

The selection loss is a measure of the generalizability of the artificial neural network (ANN), also known as its agility. Using these loss functions, one is able to optimize both the number of neurons in each hidden layer of repetitions used in the final design. In the final design of the artificial neural network (ANN) or model selection process, choose loss, also known as the error associated with the sequence and range of data, has to be taken into consideration. The output of the ANN as well as the accuracy of the output are both impacted by the amount of nodes present in the hidden layers; hence, order selection is tied to the ANN's depth. To prevent an over or underfit, it is critical to strike a balance between order selection and data complexity. The complexity of an ANN is determined by the number of hidden units as well as the node included inside those hidden layers. Using very few nodes and layers results in a higher rate of selection mistakes. In contrast, an overly complicated ANN with an excessive number of nodes or layers leads to overfitting, which raises the selection error.

It is possible to reduce the number of node and levels, and hence the complexity, of the ANN by taking steps to reduce the selection error. An ANN's selection error assesses how well it performs with fresh data when compared to its training error (generalizability). Optimizing the ANN structure needs a delicate balancing act between training and selection errors (Figure 4). In order to increase the ANN complexity, each mistake may be computed (order).

## 3. 3D CNN

The 3D CNN is a three-dimensional array of the conventional neural network, and it uses a multifiber unit like the one shown in Figure 5 and dilated weighted convolutions to extract feature attributes at different scales for volumetric segmentation.

The article "3D Convolutional Neural Network Framework with Deep Learning for Nuclear Medicine" was retracted in 2023. Reasons: signs of a paper mill; compromised peer review; unreliable results or conclusions.

*Preprocessing*: Data is preprocessed using a number of techniques before being input into the network during training (mirroring, rotation, and cropping).

*Training*: In order to train the model, we employed a patch size of 128 × 128, as well as a new loss function that merged the focused loss with the generalized loss.

*Inference*: In order for the network to properly partition the MRI data, it was zero-padded such that the original 240 × 240 × 155 voxels became 240 × 240 × 160 voxels. Once the network is ready for inference, we feed the data through it and generate probability maps. After creating these maps, the ensemble uses them to generate its given level of output.

## 4. 3D U-Net

The U-Net architecture for biomedical image segmentation was suggested in 2015 [36]. Segmenting neural structures in electron microscopy stacks or cells in light microscopy pictures proved to be a breeze for the scientists, who used the design in a number of other problems.

Convolutional layers of the U-Net design further extend this upsampling channel, enabling context information to be propagated to higher-resolution layers [36]. This creates a symmetrical U-shaped structure with a condensing and expanding route (see Figure 6). An encoder–decoder network is another name for this sort of design. For better localization, we have introduced skip links between the encoder path's high-resolution features and the decoder path's upsampled feature maps. Although U-Nets have advanced in recent years, they are still the best option for many segmentation tasks.

CNNs were often used to assign a single class label to a whole picture. However, localization is essential in many computer vision applications, where each pixel is tagged with the class of item to which it belongs. CNN classification architectures were often used for these so-called semantic segmentation problems. The classification network classifies each pixel individually by supplying a local area (also known as a patch) surrounding it. A sliding-window method is used to classify every pixel in a picture. Because so many patches can be retrieved from a single picture, this method has the added benefit of generating more training data. The restricted quantity of training data in biomedical jobs makes this particularly valuable. Although this method has its advantages, there are a few downsides. Because multiple overlapping patches need to be broadcast via the network, segmentation of a picture is a waste of time and resources. A trade-off between bigger patches providing more information and smaller ones for better localization makes it challenging to discover the ideal patch size.

The article "3D Convolutional Neural Network Framework with Deep Learning for Nuclear Medicine" was retracted in 2023. Reasons: signs of a paper mill; compromised peer review; unreliable results or conclusions.

The fully convolutional network [37] was proposed to incorporate context with high localization accuracy. Alternately, upsampling layers might be added after the normal expanding categorization network in order to get the output resolution of the picture back to where it was originally. There are no completely linked layers utilized to retain spatial data. Simple bilinear upsampling may be used to improve the output resolution. It is also possible to employ transposed convolutions, which are sometimes known as up- or deconvolutions. The transposed convolution layer's output size is determined on the kernel size and stride used.

## 5. Deep Learning's Challenges in Neuroimaging Techniques

Finally, deep learning is a kind of machine learning that employs artificial neural networks (ANN) and may be used to almost any type of learning. As a consequence, the application of deep learning to neuroimaging is still in its infancy, and various difficulties have to be addressed.

Overfitting is the one of them. Overfitting is always a problem when training a complicated classifier on a limited dataset. In general, deep learning models perform an excellent job of fitting the data, but this does not guarantee that they can be used to generalize problems. Overfitting has been reduced in several experiments by a variety of methods, including regularization [38], early halting [39], and dropping out [40]. For example, an algorithm's performance on a separate test dataset may be used to assess overfitting, but it may not perform well on comparable pictures taken at other locations, on various scanners, or with different patient demographics. In general, larger datasets from various locations are obtained utilizing various scanners and protocols with subtle differences in picture attributes, resulting in poor performance [41]. Data augmentation without standard criteria, on the other hand, cannot deal with the problems that come up when working with tiny datasets. If these technologies are to be broadly used, they must overcome a challenge known as “brittle AI.” As a result, deep learning is a data-intensive technique. In order to accomplish precise classification and confirm its performance for clinical use, a large number of well-labeled instances is needed. As opposed to classification algorithms, upstream applications like as picture quality enhancement learn from numerous predictions in a single image instead of just one (where only one learning data point is available per person). Nevertheless, the creation of large, publicly accessible medical picture datasets with labeled images is critical, notwithstanding the challenges posed by privacy issues, costs, assessing ground truth, and label accuracy [42]. Because the high dose or completely sampled pictures act as labels in the classification process, image collection applications provide an advantage over other methods because the data is already labeled. Deep learning presents a number of ethical and legal issues, as well as a problem in understanding the findings physically or mechanically. Data is fed into a “black box” and an output prediction, such as an image or classification, is generated [43]. The “Mythos of Model Interpretability” has been defined to describe the operation of all deep learning algorithms at dimensions higher than what the human mind can directly see [44]. It would be nice to get some estimates of the network's uncertainty in prediction to better understand the pictures generated.

The article "3D Convolutional Neural Network Framework with Deep Learning for Nuclear Medicine" was retracted in 2023. Reasons: signs of a paper mill; compromised peer review; unreliable results or conclusions.

It is important to realize the limitations of AI applications in the medical field, despite the fact that these applications have tremendous promise. It is well knowledge that there are challenges associated with the interpretability of models. Understanding symbolic artificial intelligence or simple convolutional neural networks, including such as regression analysis or decision trees, is still possible for humans, but it becomes extremely difficult with more advanced techniques and is now incredibly difficult with many machine learning techniques, resulting in unpredictable outcomes and nondeterministic behavior. Symbolic artificial intelligence and conventional deep learning include decision trees and linear regression. It is still unclear whether predictive AI can and should be used to make significant and important decisions when the exact mode of action is unknown, despite the fact that this problem also applies to other medical treatments (such as pharmacology in which the specific modes of action are often rarely discussed).

## 6. Conclusion

As AI has become more and more common in nuclear medicine over the last few decades, there has not been a lot of fuss or disruption. The rise of 3D CNN and U-Net applications has caused a huge shift in the landscape. From the infrazone (data and analytics) to the ultrazone (imaging), AI is being used in nuclear medicine in a wide range of ways (true synthetic intelligence). It will be easier for nuclear medicine professionals to get used to 3D CNN and U-Net for better assimilation. As a result, we think that 3D CNN and U-Net will become more and more widespread in clinical practice over the next several decades as a result of the development of explainable AI and bigger, more standardized datasets.

The article "3D Convolutional Neural Network Framework with Deep Learning for Nuclear Medicine" was retracted in 2023. Reasons: signs of a paper mill; compromised peer review; unreliable results or conclusions.

## Figures and Tables

**Figure 1:** Convolutional and pooling layer neural network.

**Figure 2:** Division of typical medical imaging workflow.

**Figure 3:** A schematic diagram of convolution and max pooling layer.

**Figure 4:** A picture of the trade-off between training and selection error.

**Figure 5:** Architecture of 3D CNN.

**Figure 6:** Architecture of 3D U-Net.

## Data Availability

No data were used for this study.
